This article has been retracted.

# Apogossypolone inhibits the proliferation of LNCaP cells *in vitro* and *in vivo*

**DOI:** 10.3892/mmr.2014.2379

**Published:** 2014-07-14

**Authors:** XIANQING ZHANG, XINGBIN HU, SHIJIE MU, YONGHUA ZHAN, QUNXING AN, ZHIXIN LIU, XIAOFENG HUANG

**Affiliations:** 1 Department of Blood Transfusion, Xijing Hospital, Fourth Military Medical University, Xi’an, Shaanxi 710032, P.R. China; 2 Engineering Research Center of Molecular and Neuroimaging, School of Life Sciences and Technology, Xidian University, Xi’an, Shaanxi 710071, P.R. China; 3 Central Laboratory, School of Basic Medicine, Fourth Military Medical University, Xi’an, Shaanxi 710032, P.R. China

**Keywords:** apogossypolone, autophagy, apoptosis, LNCaP cell, nude mouse

## Abstract

The aim of the present study was to investigate the anti-tumor effect of apogossypolone (ApoG2) on human LNCaP cells *in vitro* and *in vivo*. Cell viability was evaluated using an MTT assay. Cell autophagy and apoptosis were detected by flow cytometry and using a terminal deoxynucleotidyl transferase dUTP nick end labeling assay, respectively. Morphological autophagy alterations were observed by transmission electron microscopy. The formation of acidic vesicular organelles was assessed by acridine orange staining and fluorescence microscopy. Quantitative polymerase chain reaction (qPCR) was conducted to detect the expression levels of apoptosis-associated protein B-cell lymphoma 2 (Bcl-2) and Bak. The models of transplantation tumors in nude mice were established via subcutaneous injection of LNCaP cells. Growth of LNCaP cells was inhibited by ApoG2 treatment. Flow cytometry demonstrated that ApoG2 induced apoptosis in LNCaP cells. The Bcl-2 expression was decreased while Bak expression was increased. In addition, activation of cysteine aspartate protease (caspase)-3 and -8 was observed and 3-methyladenine (3-MA) enhanced apoptosis of LNCaP cells. Furthermore, nude mice treated with ApoG2 demonstrated a significant decrease in tumor volume and a significant increase in cell viability. Immunohistochemical analysis of tumor tissues demonstrated that ApoG2 enhanced caspase-3, -8, LC-3B and beclin-1 expression and reduced the expression of Bcl-2. ApoG2 was able to effectively suppress the growth of LNCaP cells through the induction of autophagy and apoptosis.

## Introduction

Prostate cancer, the most common neoplastic disease, is the second leading cause of cancer mortality in males. Although prostate cancers at early stages are able to be cured with surgery or radiation, other treatment options are necessary due to the high recurrence rates of this cancer (1). There are limited treatment options available for this disease. Chemotherapy and radiation therapy are largely ineffective and metastatic disease invariably recurs even following potentially curative surgery (2,3). Therefore, the development of novel anti-prostate cancer agents is required.

A novel derivative of gossypol, apogossypolone (ApoG2), has been synthesized. Compared with gossypol, ApoG2 has a higher binding affinity for anti-apoptotic Bcl-2 family proteins myeloid cell leukemia 1 and B-cell lymphoma 2 (Bcl-2) (4). Previous studies have demonstrated that ApoG2 induced significant growth inhibition *in vitro* and *in vivo*, including in a follicular small cleaved cell lymphoma model (4), lymphoma U937 cells (5), nasopharyngeal carcinoma xenografts (6) and hepatocellular carcinoma (7).

It is reported that in androgen-independent prostate cancer, members of the Bcl-2 family proteins are overexpressed (8). Whether ApoG2 has anti-tumor activity against androgen-independent prostate cancer remains to be elucidated. Apart from inducing apoptosis of tumor cells, whether ApoG2 is able to induce tumor cell death through other mechanisms is unclear. The aim of the present study was to evaluate whether ApoG2 is able to induce apoptosis and autophagy in the prostate cancer cell line LNCaP and whether it possesses anti-tumor activity in LNCaP cells in an animal model. In addition, the associated molecules involved in ApoG2-induced cell death were assessed. It was hypothesized that ApoG2 inhibits cell growth and induces autophagic cell death *in vitro*, and effectively inhibits LNCaP xenograft growth in nude mice *in vivo*.

## Materials and methods

### Materials

ApoG2, obtained from Xi’an Jiaotong University (Xi’an, China), was prepared at a stock concentration of 0.20 mmol/l in dimethyl sulfoxide (DMSO). RPMI-1640 medium, L-glutamine, trypsin-ethylenediaminetetraacetic acid, penicillin/streptomycin and fetal bovine serum (FBS) were obtained from HyClone Laboratories (Logan, UT, USA). The reagents used for the terminal deoxynucleotidyl transferase dUTP nick end labeling (TUNEL) assay were purchased from Boehringer Mannheim (Mannheim, Germany). Acridine orange was purchased from Molecular Probes (Eugene, OR, USA). Rabbit anti-LC-3B and rabbit anti-beclin-1 were purchased from Abcam (Cambridge, UK). MTT, 3-methyladenine (3-MA), annexin V-fluorescein isothiocyanate (FITC), propidium iodide (PI), Hoechst 33342, formaldehyde, HEPES, sodium pyruvate, glucose and DMSO were obtained from Sigma (St. Louis, MO, USA). All other reagents are commercially available and were of analytical grade.

### Cell culture and treatment

LNCaP cells, an androgen-independent human prostate carcinoma cell line, were obtained from the American Type Culture Collection (ATCC, Manassas, VA, USA) and cultured in RPMI-1640 supplemented with 10% FBS, 10 mmol/l HEPES, 1 mmol/l sodium pyruvate, 0.2% glucose and antibiotics. The cells were maintained at 37°C in an atmosphere of 95% air and 5% CO_2_.

For ApoG2 treatment, final concentrations of 0.01, 0.02 and 0.04 mmol/l were added and incubated for the indicated time periods. For 3-MA treatment, a final concentration of 10 mmol/l was added and incubated for the indicated time periods. For the control group, an equal volume of DMSO was added.

### MTT assay

LNCaP cell viability was assessed using an MTT assay as described by Romijn *et al* (9). Briefly, LNCaP cells were collected and resuspended in RPMI-1640 with 10% FBS and seeded into 96-well plates at a density of 5×10^5^ cells/well. Following incubation for 24 h to achieve attachment, 3-MA (10 mmol/l) and serial diluted ApoG2 (0.01, 0.02 and 0.04 mmol/l) were added. Following culturing the cells at 37°C for 24, 48, 72 and 96 h, the cells were incubated with MTT for 4 h. The plates were processed and the absorbance value was measured. Eight duplicate wells were used. The percentage of surviving cells was defined as follows: (mean absorbance of treated wells / mean absorbance of untreated wells) × 100%.

### Ultrastructural observation of LNCaP cells

The experiment was performed as described previously in PC-3 cells (10). Briefly, LNCaP cells (2×10^5^) were plated in six-well plates and incubated overnight to allow for attachment. The cells were then treated with DMSO or 0.01, 0.02 and 0.04 mmol/l ApoG2 for 24, 48, 72 or 96 h at 37°C. The cells were collected, washed twice with phosphate-buffered saline (PBS) and fixed with 2.5% ice-cold electron microscopy grade glutaraldehyde in 0.1 mol/l PBS (pH 7.3). The specimens were then rinsed with PBS and post fixed in 1% (w/v) osmium tetroxide. Following this, the specimens were dehydrated through a graded series of ethanol (30–90%) and embedded in Epon 812 resin. Using a LKB NOVA ultra-microtome (LKB, Bromma, Sweden), ultra-thin (100 nm) sections were cut and then stained with 2% (w/v) uranyl acetate and lead citrate. The sections were then examined using a JEM-2000EX transmission electron microscope (JEOL, Tokyo, Japan).

### Autophagy detection using acridine orange staining

Acridine orange staining was used to visualize the volume of the cellular acidic compartment (11). Briefly, cells were seeded in 96-well flat-bottom microtiter plates and treated as described above for the cell viability assay. At the appropriate time points following ApoG2 treatment, the cells were incubated with culture medium containing 1 mg/ml acridine orange for 15 min. The acridine orange was removed and fluorescent micrographs were captured using a DM-IRB inverted fluorescent microscope (Leica, Wetzlar, Germany). For each experiment condition, autophagy was quantified based on the mean number of cells exhibiting intense red staining in three fields (containing at least 50 cells per field).

### Autophagy analysis by flow cytometry

The percentage of autophagic cell death was analyzed using flow cytometry as previously described (11). Briefly, the cells were treated with DMSO (control) or 0.01, 0.02 and 0.04 mmol/l ApoG2 for 48 h at 37°C. The cells were then stained with acridine orange for 20 min. The adhering cells and the suspending cells in the medium were collected in phenol red-free RPMI-1640 medium. The fluorescence emission of green and red was measured using a flow cytometer (FACSAri; Becton Dickinson, Mountain View, CA, USA) using CellQuest software (BD Biosciences San Jose, CA, USA). The percentage of autophagy was calculated by adding the values from the upper-left and upper-right quadrants. 3-MA was added to detect its effect on ApoG2-induced cell death. The cells were treated with 10 mmol/l 3-MA and 0.02 mmol/l ApoG2 for 48 h and the percentage of autophagic cell death was analyzed as described above.

### Apoptosis analysis by flow cytometry

Apoptosis was analyzed by annexin V/propidium iodide (PI) staining according to a previous study (10). In brief, LNCaP cells were treated with DMSO or 0.01, 0.02 and 0.04 mmol/l ApoG2 for 24, 48, 72 and 96 h at 37°C. The cells were trypsinized and washed in cold PBS. Subsequently, the cells were stained with FITC-labeled annexin V and PI for 15 min and were then analyzed by flow cytometry. The percentage of apoptosis was calculated by the addition of primary apoptosis (annexin V+/PI−) and late apoptosis (annexin V+/PI+).

### Apoptosis analysis using the TUNEL assay

The TUNEL assay was performed according to the manufacturer’s instructions. Briefly, following treatment with 0.02 mmol/l ApoG2 and 10 mmol/l 3-MA, the cells were fixed. The cells were then washed, stained and images were captured using the Olympus FV1000 laser scanning confocal microscope (Olympus, Tokyo, Japan). Treatment with DNaseI prior to TUNEL staining was used as a positive control. For quantitative analysis, the percentage of TUNEL-positive cells among 200 cancer cells in three visual fields per section was determined (magnification, ×200).

### Cell cycle analysis by flow cytometry

The cells were processed for cell cycle analysis 48 h after ApoG2 treatment. Briefly, cells (1×10^6^/ml) were fixed in chilled methanol overnight prior to staining with 50 mg/ml PI, 1 mg/ml RNase and 0.1% NP40. Analysis was performed immediately following staining using a FACSAri flow cytometer (Becton Dickinson). All experiments were independently performed at least three times.

### Immunofluorescence

LNCaP cells (1×10^5^) were grown on cover slips and incubated overnight to allow for attachment. Then, cells were treated with ApoG2 for the desired time period at 37°C, washed with PBS and fixed at 4°C overnight using 4% paraformaldehyde. Subsequently, the cells were washed with PBS and blocked with PBS containing 0.5% bovine serum albumin (BSA) and 0.15% glycine (BSA buffer) for 1 h at room temperature. Finally, the cells were labeled with primary antibodies (rabbit anti-human anti-LC-3B monoclonal antibody and rabbit anti-human anti-beclin-1 monoclonal antibody; Abcam) and secondary antibodies (FITC-conjugated goat anti-rabbit polyclonal antibody; Abcam) for 1 h at room temperature, respectively. In negative controls, the primary antibodies were omitted. For fluorescence observation, the slides were examined under an Olympus fluorescence microscope.

### Analysis of cysteine aspartate protease (caspase)-3 and caspase-8 activity

Caspase-3 and caspase-8 activities were detected according to the manufacturer’s instructions of the caspase colorimetric assay kit (Sigma). Briefly, cells (10^8^ cell/ml) were collected and resuspended in ice-cold buffer. Following lysis, cell lysates were centrifuged at 12,000 × g for 10 min and the extracts containing 50 μg of protein were incubated with 100 μl of Ac-DEVD-pNA substrate at 37°C for 2 h. The colorimetric release of p-nitroaniline from the Ac-DEVD-pNA substrate was measured at 405 nm.

### Semi-quantitative reverse transcription-polymerase chain reaction (RT-PCR)

The cells were collected and TRIzol extraction of total RNA was performed 48 h after ApoG2 treatment according to the manufacturer’s instructions (Qiagen GmbH, Hilden, Germany). Semi-quantitative RT-PCR was performed using the RNA PCR kit. The following PCR procedures were used: pre-denaturation at 94°C for 3 min, 30 cycles of 95°C 30 sec, 57°C 30 sec, 72°C 1 min and a final extension at 72°C for 1 min. The primer pairs used are shown in Table I. GAPDH was used as an internal control. The PCR products and DNA marker were run on ethidium bromide-stained 1.5% agarose gels in tris-borate-EDTA. Images were acquired and quantification of the bands was performed by image analysis software for Gel Electrophoresis samples. Band intensity was expressed as relative absorbance units. Following normalization to GAPDH, the mean value and the standard deviation were calculated.

### Western blotting

The cells were lysed for western blot analysis 48 h after ApoG2 treatment. Cell lysates were resolved by 10% sodium dodecyl sulfate polyacrylamide gel electrophoresis and electrotransferred onto nitrocellulose membranes. Membranes were blocked with 5% dry milk in PBS-Tween for 1 h at room temperature and then incubated with the primary antibodies overnight at 4°C. Primary antibodies included mouse anti-human anti-Bcl-2 (1:1,000) and mouse anti-human anti-Bak monoclonal antibodies (1:500; Abcam). Additionally, β-actin was used as an internal control. Following incubation with primary antibodies, the membranes were washed and incubated with horseradish peroxidase-labeled secondary antibodies for 1 h at room temperature. The membranes were subsequently incubated with the ECL for 1 min and autoradiographed using X-ray film.

### Animals and experimental design

Male BALB/c nude mice (4 weeks old, weighing 18–22 g) were purchased from the Laboratory Animal Center of the Fourth Military Medical University (Xi’an, Shaanxi, China). They were kept in standard conditions. A total of 40 mice were injected with 1.0×10^7^ LNCaP cells subcutaneously on the two sides of the lower back above the tail. Palpable tumors (volume 200 mm^3^) were formed following 7 days and the mice were randomly divided into four groups, including the negative control group and the 2.5, 5.0 and 10.0 mg/kg ApoG2 treatment groups. The negative control group received 0.9% normal saline containing 1% DMSO. All of these drugs were injected intraperitoneally daily up to 30 days. The tumor size was measured once every 2 days in two perpendiculars and tumor volume (TV) was calculated using the following formula: (ab^2^) / 2, where a and b refer to the longer and shorter dimension, respectively (12). A technician from the Laboratory Animal Center of the Fourth Military Medical University measured the tumor sizes and animal body weights daily without knowledge of the treatment. All animal experiments were performed according to the protocol approved by the Fourth Military Medical University Guidelines for the Use and Care of Animals. Tumor growth inhibition (T/C%) values for these *in vivo* studies were calculated as described previously (13). If the mouse died, the transplanting tumor and its liver, kidney, heart and intestines were removed for histological analysis. The tissues were fixed overnight in 4% paraformaldehyde in PBS and embedded in paraffin. Sections (5 μm) were deparaffinized, rehydrated and stained with hematoxylin and eosin (H&E). The tumor growth inhibition rate was calculated using the following formula: inhibition rate (%) = (mean tumor weight of negative control group - mean tumor weight of treatment group) / mean tumor weight of the negative control group.

### Immunohistochemistry

The expression levels of Bcl-2, CD31, caspase-3, caspase-8, LC-3B and Beclin-1 in tumor tissues were detected by immunohistochemistry. Briefly, tumor tissues were embedded in paraffin. Sections (5 μm) were deparaffinized, rehydrated and blocked for 1 h at room temperature. Following labeling with primary and secondary antibodies, slides were mounted and examined under an Olympus fluorescence microscope. In negative controls, the primary antibodies were omitted. The fluorescence intensity of each protein was semi-quantitatively analyzed using ImagePro Plus 6.0 software (Media Cybernetics, Silver Spring, MD, USA). Five visual fields in each section were selected for the determination of the integrated fluorescence intensity and area. The expression level was represented by the integrated fluorescence intensity per unit area.

### Microvessel density (MVD) assessment

Using a two-headed microscope, immunohistochemical reactions for CD31 antigen were independently interpreted by two authors. Within the tumor, the two most vascularized areas (‘hot spots’) were selected (magnification, ×10) and the vessels were counted in a representative high magnification (x200) field in each of these two areas. Next, the high-magnification fields were marked for subsequent image cytometric analysis. Single immunoreactive endothelial cells or endothelial cell clusters that were separate from other microvessels were counted as individual microvessels. Mean visible microvessel density for CD31 was calculated as the average of five counts.

### Statistical analysis

SPSS version 11.0 (SPSS, Inc., Chicago, IL, USA) for Windows was used for all statistical analyses. All data are presented as the mean ± standard deviation. Analysis of variance followed by the Tukey test or Dunnett’s test were used to analyze the significance of any difference among groups. P<0.05 was considered to indicate a statistically significant difference.

## Results

### ApoG2 inhibits the growth of LNCaP cells

To determine the effect of ApoG2 on cell viability in LNCaP cells, the cells were initially treated with ApoG2 (0.01, 0.02 and 0.04 mmol/l) and cell viability was measured using the MTT assay. Compared with the control cells (Fig. 1A), cell viability in cells treated with ApoG2 was significantly lower (^*^P*<*0.05 and ^**^P<0.01). In addition, ApoG2 inhibited the growth of LNCaP cells in a dose-dependent manner. However, when cells were treated with ApoG2 and 3-MA, cell viability was significantly decreased (Fig. 1A). Notably, ApoG2 also inhibited the growth of LNCaP cells in a time-dependent manner (Fig. 1B). The inhibition pattern of ApoG2 was similar to that in Fig. 1A. Furthermore, 3-MA aggravated the inhibitory effect of ApoG2. Following treatment for 72 h with ApoG2, the IC_50_ was 0.009 mmol/l (Fig. 1). IC_50_ values were calculated using the CelTox software available from Aniara Corporation (Mason, OH, USA). These results indicated that ApoG2 inhibited the growth of LNCaP cells in a time- and dose-dependent manner.

### Characteristic autophagic alterations at the ultrastructural level induced by ApoG2

To determine whether ApoG2 was able to induce autophagy, the ultrastructural alterations of LNCaP cells were observed under a JEM-2000EX transmission electron microscope (JEOL Ltd., Tokyo, Japan). In untreated cells, no autophagic vacuoles were observed and clear microvilli were observed on LNCaP cell surfaces, with euchromatin-dominant nuclei and clear nucleoli (Fig. 2A). However, following treatment with ApoG2, characteristic autophagic morphological alterations were observed. Surface microvilli were decreased, numerous autophagic vacuoles were observed and the vacuoles were packed with membrane structures and cell debris (Fig. 2B). This result suggested that ApoG2 was able to induce autophagy in LNCaP cells.

### ApoG2 induces apoptosis and cell cycle arrest in LNCaP cells

To investigate the effect of ApoG2 on apoptosis, flow cytometry and a TUNEL assay were performed. Flow cytometric results (Fig. 3A) demonstrated that the apoptotic rate was 2.8, 8 and 11.1% at 0.01, 0.02 and 0.04 mmol/l of ApoG2 treatment and that the apoptotic rate was 40.6% when cells were treated with ApoG2 and 3-MA. The increase in the apoptotic rate was significant (^*^P<0.05 and ^**^P<0.01). These data suggested that ApoG2 was able to induce apoptosis in a dose-dependent manner and inhibition of autophagy was able to increase the apoptosis of LNCaP cells. This result was further verified using a TUNEL assay. TUNEL-positive nuclei in ApoG2-treated LNCaP cells (Fig. 3B) was similar to that in the control, whereas TUNEL-positive nuclei in cells treated with ApoG2 and 3-MA were significantly increased (^*^P<0.05 and ^**^P<0.01). Quantitative results are shown in Fig. 3C. In the control cells, the apoptotic rate (1.2±0.1%) was lower than that in cells treated with ApoG2 (3.2±0.3%). However, the difference between the two groups was not significant (P>0.05). When cells were treated with ApoG2 and 3-MA, the percentage of apoptotic cells induced by ApoG2 increased up to 45.6±1.4%. Compared with the ApoG2 only group, the apoptotic rate induced by 3-MA and ApoG2 was significantly increased (P<0.01).

Next, the effect of ApoG2 on the cell cycle distribution of LNCaP cells was analyzed. As shown in Fig. 3D, a clear subG1 peak was identified, suggesting that the percentage of apoptotic cells induced by ApoG2 was increased with the increase in ApoG2 concentration. The number of cells in the G1 phase was also increased following treatment with ApoG2. The percentage of cells in the G1 phase was 60% in the control, whereas it was increased to 65–80% following treatment with ApoG2. In addition, along with the increasing concentration of ApoG2, the percentage of cells in the S phase decreased. Furthermore, a significant decrease in cells in the S phase was noted following treatment with 0.02 mmol/l ApoG2. ApoG2 resulted in a dose-dependent cell cycle arrest in the G0/G1 phase.

### Expression of Bcl-2 and Bak at the mRNA and protein level

RT-PCR was performed to investigate the effect of ApoG2 on Bak and Bcl-2 mRNA expression (data not shown). The mRNA expression level of Bcl-2 (Bcl-2/GAPDH value 0.429) in ApoG2-treated LNCaP cells was lower than that in the control cells (Bcl-2/GAPDH value 0.6267). By contrast, the mRNA expression level of Bak (Bak/GAPDH value 0.4743) was higher in ApoG2-treated LNCaP cells than in the control cells (Bak/GAPDH value 0.2667). The expression levels of Bak and Bcl-2 at the protein level were detected by western blot analysis (Fig. 4A). At 24 h after ApoG2 treatment, the expression level of the Bcl-2 protein in ApoG2-treated LNCaP cells was similar to that in the control cells. However, 48 and 72 h after ApoG2 treatment, the expression level of Bcl-2 protein in ApoG2-treated cells was lower than that in the control cells. Similarly, 24 h after ApoG2 treatment, the expression level of the Bak protein in ApoG2-treated LNCaP cells was similar to that in the control cells. While at 48 and 72 h after ApoG2 treatment, the expression level of the Bak protein in ApoG2-treated LNCaP cells was higher than that in the control cells. These data demonstrated that the expression level of the anti-apoptotic protein Bcl-2 was decreased while the expression level of pro-apoptotic protein Bak was increased.

### Caspase-3 and caspase-8 are activated in ApoG2-treated cells

Caspases, a family of cysteine proteases, have a central role in the execution of apoptosis. To examine whether ApoG2 induces apoptosis through the activation of caspases, a colorimetric substrate Ac-DEVD-pNA for caspases was used to detect caspase activity. As shown in Fig. 4B, the activity of caspase-3 and caspase-8 in LNCaP cells treated with ApoG2 was significantly higher than that in the control cells. This suggested that ApoG2 induced apoptosis by triggering the activation of caspase cascades.

### ApoG2 induces the formation of acidic vesicular organelles (AVOs) in LNCaP cells

Formation of AVOs is another characteristic feature of cells engaged in autophagy (2,11). Therefore, the effect of ApoG2 treatment on the formation of AVOs in LNCaP cells following acridine orange staining was assessed (Fig. 5A). Acridine orange is a weak base that has the ability to move freely across biological membranes in an uncharged state and is characterized by green fluorescence. Acridine orange, in its protonated form, accumulates in acidic compartments and forms aggregates, which are characterized by red fluorescence. As shown in Fig. 5A, control LNCaP cells primarily exhibited green fluorescence, indicating a lack of AVOs. By contrast, treatment of LNCaP cells with ApoG2 induced the formation of red fluorescent AVOs. In addition, compared with the 0.01 mmol/l ApoG2 treatment group, the red fluorescent AVOs were more marked at 0.02 and 0.04 mmol/l of ApoG2 treatment. These results were consistent with the flow cytometric results and provided further evidence to indicate that ApoG2 treatment caused autophagy in LNCaP cells.

### ApoG2 induces the expression of Beclin-1 and LC-3B protein in LNCaP cells

LC-3B reflects autophagic activity and detecting LC-3B by immunofluorescence has become a reliable method for monitoring autophagy. Beclin-1 is important in autophagy and is involved in the formation of autophagosomes. The immunofluorescence results demonstrated that in the control cells, no clear Beclin-1 and LC-3B expression was observed. However, in LNCaP cells treated with ApoG2, Beclin-1 (Fig. 5B) and LC-3B (Fig. 5C) expression exhibited a punctate pattern. These results indicated the presence of autolysosomes or autophagolysosomes in LNCaP cells following treatment with ApoG2 (14).

### Autophagy detection with acridine orange staining and flow cytometry

The fluorescence of the cytoplasm and nucleolus was bright green and dim red in acridine orange-stained cells, whereas the acidic compartments were characterized by bright red fluorescence (15). Thus, the intensity of the red fluorescence was proportional to the degree of acidity. Therefore, the volume of the cellular acidic compartment was able to be quantified (16). To further quantify the formation of AVOs in LNCaP cells, acridine-stained cells were analyzed by flow cytometry. Quantitative results are shown in Fig. 5D. The percentage of AVOs in 0.01, 0.02 and 0.04 mmol/l ApoG2 treatment groups was 13.7, 28.9 and 51.8%, respectively. When the cells were treated with 3-MA and ApoG2, the ratio of AVOs in LNCaP cells decreased to 3.2%. This result further confirmed that ApoG2 treatment was able to induce autophagy in LNCaP cells.

### Effects of ApoG2 on tumor growth and animal survival rate

Tumor volumes were recorded every 2 days until day 10. On day 4, tumor volumes in the 5.0 and 10.0 mg/kg ApoG2 treatment groups were significantly decreased. On day 10, there was a 6.5-fold increase in tumor volumes in the control group. However, the elevation in tumor volumes in the ApoG2 treatment groups was 2.5-fold (10.0 mg/kg), 3.7-fold (5.0 mg/kg) and 4.8-fold (2.5 mg/kg), respectively (Fig. 6A).

The tumor growth inhibition (T/C%) ratio was calculated as previously described (13) and is summarized in Table II. According to the National Cancer Institute (NCI) criteria, a reagent with a T/C% <42% is considered to have significant anti-tumor activity. A reagent with a T/C% <10% is considered to have highly significant anti-tumor activity and this is also the criteria used by the NCI to justify a clinical trial (12). The T/C% in the 10 mg/kg ApoG2 treatment group was 21.3%, indicating that ApoG2 possesses significant anti-tumor activity.

All the nude mice with xenografts died after 16 days. As shown in Fig. 6B, the survival rate of the 10.0 mg/kg group was 20% on day 21. The survival rate of the 5.0 mg/kg group was 80% on day 26 and the survival rate of the 2.5 mg/kg group was 20% at the end of the experiment. The Log-rank inspection analysis demonstrated a significant difference between the survival rates of the animals at different doses of ApoG2 when compared with the control group.

### Histopathological features of transplanted tumors

The histopathologic alterations of transplanted tumor were analyzed by H&E staining. As shown in Fig. 7A, areas of necrosis were not observed in the control group. However, the percentage of cells undergoing necrosis in the three ApoG2 groups (2.5, 5.0 and 10.0 mg/kg) was 3.5±0.3, 20.3±2.5 and 53.3±3.6% of total nucleated cells, respectively.

### Histopathological features of the liver and intestine in ApoG2-treated mice

In order to determine whether ApoG2 had a toxic effect in other organs, the histopathological changes of the liver and intestine were observed by H&E staining. As shown in Fig. 7B, in the 10.0 mg/kg ApoG2 treatment group there was partial pathological alterations with spotty necrosis, inflammatory cell infiltration and integral hepatic lobule in the liver. In the 5.0 and 2.5 mg/kg ApoG2 treatment group no significant pathological alterations in the liver were observed.

A similar pattern was observed in the intestine (Fig. 7C). An integral intestinal mucosa structure and normal epithelial cells were observed in the 10.0 mg/kg ApoG2 treatment group in the small intestine. While no significant pathological changes were observed in the small intestine in the 5.0 and 2.5 mg/kg ApoG2 treatment groups.

These results indicated that the ApoG2 doses used in the present study do not have toxic effects on the liver and intestine.

### Expression of caspase-3 and caspase-8 in tumor tissues

As mentioned above, caspase-3 and caspase-8 were activated in ApoG2-treated LNCaP cells. Furthermore, whether caspase-3 and caspase-8 were activated in tumor tissues was analyzed. As shown in Fig. 8A and B, the expression levels of caspase-3 and caspase-8 were extremely low and hardly detectable in the negative control group. However, following treatment with ApoG2, the expression levels of caspase-3 and caspase-8 were increased. Compared with the negative control group, significant differences in the 10.0 mg/kg ApoG2 treatment group were identified for caspase-3 (Fig. 8A) and in the 5 and 2.5 mg/kg ApoG2 treatment group for caspase-8 (Fig. 8B). These data suggested that tumor tissue underwent apoptotic cell death following ApoG2 treatment.

#### Expression of Bcl-2, Beclin-1 and LC-3B in tumor tissues in vivo

As revealed by RT-PCR and western blot results (Fig. 4A), Bcl-2 expression levels were downregulated in ApoG2-treated LNCaP cells. Immunohistochemistry for Bcl-2 was performed to determine whether this was also the case in tumor tissues. As shown in Fig. 8C, the Bcl-2 fluorescent intensity in ApoG2-treated cells were only partially decreased. No significant difference was identified among the control group and the ApoG2 treatment group. This result indicated that the impact of ApoG2 on the expression of Bcl-2 in human prostatic cancer xenograft tissues was not significant.

As shown in Fig. 5, ApoG2 induced the expression of Beclin 1 and LC-3B in LNCaP cells *in vitro*. In fact, this was also true in tumor tissues *in vivo*. In the control group, Beclin 1 and LC-3B fluorescence intensity were extremely low. However, following treatment with ApoG2, the fluorescence intensity of Beclin 1 (Fig. 8D) and LC-3B (Fig. 8E) increased in a dose-dependent manner. Compared with the control group, the Beclin 1 and LC-3B fluorescence intensity of the ApoG2 treatment group were significantly higher.

### ApoG2 affects the angiogenesis of tumor tissues

To evaluate the effect of ApoG2 on the angiogenesis of tumor tissues, MVD was analyzed by labeling CD31, which was expressed in the cytoplasm of vascular endothelial cells. As shown in Fig. 8F, CD31 expression in tumor tissues of the control group was clear and connected into a network. However, the expression of CD31 in tumor tissues of ApoG2 treatment groups decreased by various degrees. The decrease in CD31 expression in the 10.0 mg/kg ApoG2 treatment group was most marked. In addition, the decrease in CD31 expression of the 5.0 mg/kg ApoG2 treatment group was also significant. In the 2.5 mg/kg ApoG2 treatment group, CD31 expression remained clear but with decreased vessel density, suggesting that these vessels were not connected into a network. The MVD count analysis demonstrated that the MVD in each ApoG2 treatment group was significantly smaller than that of the negative control group (Fig. 8F). These data suggested that angiogenesis was impaired in ApoG2-treated tumor tissues.

## Discussion

Prostatic cancers are a type of malignant tumor that endanger the health of males. The incidence rate of prostate cancer in America has exceeded lung cancer and its mortality rate is in second place to lung cancer (1). Furthermore, the incidence rate and the morality rate of the prostatic cancers also show an increasing trend year after year. There are various methods used for the treatment of prostatic cancer, including surgery, chemotherapy, endocrine therapy and immune therapy. Among them, endocrine therapy is an important and essential method for the treatment of prostatic cancer, which may prolong the survival time of patients with terminal prostatic cancer. However, due to steroid resistance or transfer, the conditions of a considerable number of patients still worsen, leading to mortality. Therefore, the investigation and development of new agents with high efficiency and low toxicity has drawn the attention of scientists, particularly scientists in the field of phytochemistry. The levorotation gossypol is a natural product derived from the seeds and roots of cotton and has been used as male contraceptive drugs for >30 years in China (17). In 1984, Tuszynski *et al* (18) revealed that gossypol had anti-tumor activity against melanoma and colorectal cancer. Since then numerous studies have reported the anti-proliferation activity of the gossypol against tumor cells, including colon cancer cells (19), head cervical squamous carcinoma cells (20), diffuse large cell lymphoma cells (21) and prostatic cancer cells (22). However, the gossypol may result in larger toxic side effects. The stable Schiff’s alkali is easily formed between the two chemically active aldehyde groups of the gossypol and the amino acid residues of the proteins. ApoG2 is the derivative of the gossypol with the two aldehyde groups removed. It was able to inhibit Bcl-2 and have a higher anti-tumor activity than the gossypol (23).

The present study found that the tumor volume of the tumor-bearing mice was significantly smaller than that of the control group following ten days treatment with ApoG2. Furthermore, no weight loss occurred during the treatment, demonstrating that the ApoG2 dosage used in the present study was not toxic to the animals. Additionally, the histopathological examination results demonstrated that the animals had no heart and kidney injuries following consecutive 23 days treatment with ApoG2. The hepatic and intestinal toxicity was extremely small and significantly lower than the (−) - gossypol (data not shown). Therefore, ApoG2 had improved tumor specificity. All the results indicate that ApoG2 may be a safe and effective drug for the treatment of prostatic cancer.

It is reported that autophagy is important in the development of tumor and that the autophagosome degradation capacity of the tumor cells is smaller than that of normal cells (24). Several studies have demonstrated that in mammals autophagy may interact with apoptosis under certain conditions (25,26). Autophagy is possibly one of the prerequisites of apoptosis. It occurs prior to apoptosis and may enhance the activity of the latter. By contrast, autophagy and apoptosis may be subjected to the antagonist effect or inter-conversion (27–29). The association between the two cell death pathways, including the effect of apoptotic deficiencies on autophagy requires further investigation. Our experimental data demonstrated that, following the effect of ApoG2, LNCap cells exhibited clear characteristics of autophagy, including the appearance of membranous vacuoles in the cytoplasm and formation of AVOs, as well an increase in the expression of the autophagy-associated proteins LC-3B and beclin 1. In addition, 3-MA, a phosphatidylinositol 3-kinase inhibitor, which is commonly used as a specific inhibitor of autophagic sequestration, increased cell apoptosis, demonstrating that autophagy and apoptosis may convert with each other under certain conditions. The present study reported that ApoG2 induced apoptotic and autophagic cell death in LNCaP cells. The pro-apoptotic proteins (including Bak, Bax and Bad) and autophagic proteins may all merge with the same area of Bcl-2/Bcl-XL. Therefore, it may be inferred that ApoG2 simultaneously induces autophagic cell death and apoptotic cell death of LNCap cells, making ApoG2 an attractive molecular tool to investigate the association between autophagic cell death and apoptotic cell death.

In conclusion, data from the present study demonstrated that ApoG2 may significantly inhibit the growth of LNCaP cells through inducing autophagic cell death and that ApoG2 may be a potentially effective chemical drug for the treatment of prostatic cancer.

## Figures and Tables

**Figure 1:** Effect of ApoG2 on cell viability in LNCaP cells. Cell viability was measured by the MTT assay. (A) LNCaP cells were treated with ApoG2 (0.01, 0.02 and 0.04 mmol/l) or 3-MA (10 mmol/l) for 24 h prior to the MTT assay. ^*^P<0.05. ^**^P<0.01, compared with the control. (B) LNCaP cells were treated with 0.02 mmol/l ApoG2 and 10 mmol/l 3-MA for 24, 48, 72 and 96 h prior to the MTT assay. The percentage of surviving cells was defined as (mean absorbance of treated wells / mean absorbance of untreated wells) × 100%. All results are expressed as the mean ± standard error of the mean of three independent experiments. ^*^P<0.01, compared with the 0 h group. ApoG2, apogossypolone; 3-MA, 3-methyladenine.

**Figure 2:** Ultra-structural alterations in LNCaP cells analyzed using a transmission electron microscope. LNCaP cells were seeded in culture bottles and treated (A) without or (B) with 0.02 mmol/l ApoG2 for 24 h.

**Figure 3:** Apoptosis and cell cycle distribution analysis. (A) Flow cytometric analysis of cell apoptosis. LNCaP cells were treated with 0.01, 0.02 and 0.04 mmol/l ApoG2 and 0.02 mmol/l ApoG2 + 10 mmol/l 3-MA for 48 h, respectively. Then, cells were collected and stained with fluorescein isothiocyanate-Annexin V to detect cell apoptosis by flow cytometry. Quantitative results are shown. (B) Cell apoptosis measured using a terminal deoxynucleotidyl transferase dUTP nick end labeling assay. Representative images were captured at a magnification of ×200. (C) Quantitative results of the apoptotic rate in (B). (D) Cell cycle distributions of ApoG2-treated LNCaP cells analyzed by flow cytometry. The cells were treated with dimethyl sulfoxide and 0.01, 0.02 and 0.04 mmol/l ApoG2 for 48 h. All results are expressed as the mean ± standard error of the mean of three independent experiments. ^*^P<0.05 and ^**^P<0.01 compared with the negative control group. ApoG2, apogossypolone.

**Figure 4:** Analysis of apoptosis-associated proteins Bcl-2, Bax, caspase-3 and caspase-8. (A) Western blot analysis of expression of Bak and Bcl-2 proteins in LNCaP cells treated with 0.02 mmol/l ApoG2 for indicated times. (B) Caspase activity assay. The cells were treated with ApoG2 prior to analysis. All results are expressed as the mean ± standard error of the mean of three independent experiments. ^*^P<0.05 and ^**^P<0.01 compared with the control. Bcl-2, B-cell lymphoma-2; caspase, cysteine aspartate protease; ApoG2, apogossypolone.

**Figure 5:** Autophagy analysis by acridine orange staining and expression levels of beclin-1 and LC-3B by immunocytochemistry. The cells were treated with ApoG2 or ApoG2 and 3-MA for 48 h prior to analysis. (A) Acridine orange staining results. (B) Expression of beclin-1. (C) Expression of LC-3B. (D) Quantitative flow cytometry results of autophagy. ^*^P<0.05, compared with the control. ApoG2, apogossypolone; 3-MA, 3-methyladenine.

**Figure 6:** Effects of ApoG2 on the tumor volume and survival rate of athymic nude mice bearing LNCaP cells. (A) Tumor volume of control and ApoG2 treatment groups. All results are expressed as the mean ± standard error of the mean of three independent experiments. (B) Survival rate of athymic nude mice in the control and ApoG2 treatment groups. ApoG2, apogossypolone.

**Figure 7:** Effects of ApoG2 on the pathological features of transplanted tumors, liver and intestine. (A) Transplanted tumors (H&E; magnification, ×400). (B) Liver (H&E; magnification, ×400). (C) Intestine (H&E; magnification, ×400). H&E, hematoxylin and eosin; ApoG2, apogossypolone.

**Figure 8:** Immunohistochemical analysis of caspase-3, caspase-8, Bcl-2, LC-3B, Beclin 1 and CD31 in tumor tissues. The LNCaP xenograft was treated with ApoG2 for 10 days. Representative immunohistochemical results are shown. (A) Expression of caspase-3 (magnification, ×400). (B) Expression of caspase-8 (magnification, ×400). (C) Expression of Bcl-2 (magnification, ×400). (D) Expression of LC-3B (magnification, ×400). (E) Expression of beclin 1 (magnification, ×400). (F) Expression of CD31 (magnification, ×400). All results are expressed as the mean ± standard error of the mean of three independent experiments. Bcl-2, Bcl-2, B-cell lymphoma-2; ApoG2, apogossypolone; caspase, cysteine aspartate protease.

**Table I:** Primers used in the present study.

Gene	Primer	Primer sequence
Bcl-2	Bcl-2F	5′-gagttcgccgagatgtccag-3′
	Bcl-2R	5′-tcacttgtggctcagatagg-3′
Bak	BakF	5′-acgctatgactcagagttcc-3′
	BakR	5′-cttcgtaccacaaactggcc-3′
GAPDH	GAPDH_F	5′-acatcgctcagacaccatgg-3′
	GAPDH_R	5′-gtagttgaggtcaatgaaggg-3′

Bcl-2, B-cell lymphoma 2; F, forward; R, reverse.

**Table II:** Comparison of tumor growth inhibition (T/C%) versus initial tumor sizes in the *in vivo* experiments.

Group	Initial tumor size (cm^3^)	T/C%
Control	0.220	100.0
ApoG2 2.5 mg/kg	0.231	82.1
ApoG2 5.0 mg/kg	0.225	67.9
ApoG2 10.0 mg/kg	0.228	21.3

Tumor growth inhibition (T/C%) was calculated as the percentage median tumor size in the treatment group versus the control group.
